This article has been retracted.

# To Summarize and Analyze the Epidemiological Characteristics and Prognostic Risk Factors of Patients with Pelvic Fracture Complicated with Perineal Injury

**DOI:** 10.1155/2022/4831330

**Published:** 2022-03-30

**Authors:** Wen Li, Shasha Du, Houcai Guo, Xuan Han, Tao Huang

**Affiliations:** ^1^General Hospital of Central Theater Command, No. 627 Wuluo Road, Wuhan, Hubei Province 430070, China; ^2^Daye City People's Hospital, No. 25 Dongfeng Road Chengbei Development Zone, Daye, Hubei Province 435100, China

## Abstract

This study is aimed at summarizing and analyzing the epidemiological characteristics and prognostic risk factors of patients with a pelvic fracture with perineal injury. The clinical data of 153 patients with pelvic fracture with perineal injury treated in our hospital from January 2012 to June 2021 were analyzed retrospectively. The data of sex, age, injury mechanism, pelvic fracture type, shock index (SI), perineal wound depth, concomitant injury, total hospital stay, and death were collected by the electronic medical record system. Among the 153 patients, there were 94 males and 59 females, with an average age of (43.2 ± 16.8) years. The cases were mainly concentrated into two age groups: 20–29 years old and 50–59 years old. In a year, pelvic fractures were mainly concentrated in 1–2 months and 11–12 months. In terms of injury time, there were mainly two periods of time in a day: 10 : 00～12 : 00 and 15 : 00～18 : 00. The MOTS-RTS scores of the patients in the undead group and the dead group were (7.12 ± 1.52), (2.69 ± 0.96), ISS scores were (27.36 ± 15.84), (61.32 ± 7.08), GCS scores were (12.84 ± 3.69), (4.13 ± 1.25), APACH II scores were (12.87 ± 8.84), (32.41 ± 6.98), and SOFA scores were (6.68 ± 5.87), (17.12 ± 3.12). The MOTS-RTS and GCS scores of the nondeath group were significantly higher, while the ISS score, APACH II score, SOFA score, and shock index were significantly lower. The overall mortality rate of 153 patients was 13.7%. The average area of perineal trauma in undead and dead patients was (54.5 ± 113.52) cm^2^ and (262.63 ± 300.84) cm^2^, respectively. The average depth of perineal trauma was (9.63 ± 7.22) cm and (16.23 ± 10.13) cm, respectively. The larger the area of perineal injury and the deeper the depth of perineal trauma, the worse their prognosis. Cox multivariate analysis showed that complications, MOTS-RTS score, ISS score, GCS score, perineal trauma area, and perineal trauma depth were independent risk factors affecting the prognosis of patients with pelvic fracture with perineal injury. Most of the patients with pelvic fracture complicated with perineal injury are 20–29 years old and 50–59 years old. The more serious the perineal injury is, the higher the mortality is. The main causes of death are refractory hemorrhagic shock and infection.

## 1. Introduction

About 10% of pelvic fractures are unstable pelvic fractures, which are often caused by high-energy injuries such as car accidents, fall injuries, and crush injuries [1]. From the mechanical point of view, the severity of the injury is mainly related to the magnitude and direction of the external force, the location of the focus, and the inertia of the patient [2]. Pelvic fractures are often accompanied by injuries of the abdomen, pelvic organs, urinary system, retroperitoneal nerves, and vessels. The main types of concomitant injuries include traumatic pelvic fracture, laceration or absence of external genitalia, anorectal laceration, urethral contusion, and urethral rupture [3]. Pelvic fracture often leads to an injury of important organs in the abdominal cavity, and the mortality rate is significantly higher in the case of improper diagnosis and treatment [4]. The disability rate and mortality rate of unstable pelvic fracture were high. The main cause of death within 24 hours was fatal bleeding, while organ injury, brain injury, and/or multiple organ failure were the main causes of death 24 hours later [5]. Due to the vast territory of our country, there are great differences in socioeconomic development and population composition in different regions; the patients treated in different levels of hospitals are different, and the results of epidemiological studies on pelvic trauma are also different [6]. At present, there are many literature reports on the emergency treatment of patients with pelvic fracture, and a wealth of experience has been accumulated, but it focuses on the treatment time, surgical methods, related laboratory tests including blood transfusion, and the effect of each operation [7]. There are a few studies on the epidemiological characteristics of patients with pelvic fracture. Our paper analyzed the relevant data of patients with pelvic trauma in this area, in order to provide a basis for more efficient prevention and treatment for this kind of injury.

## 2. Materials and Methods

### 2.1. Patient Data

The clinical data of 153 patients with a pelvic fracture with perineal injury treated in our hospital from January 2012 to June 2021 were analyzed retrospectively. The data of sex, age, injury mechanism, pelvic fracture type, shock index (SI), major trauma outcome study-revised trauma score (MOTS-RTS), injury severity score (ISS), Glasgow coma scale (GCS), acute physiology and chronic health score (APACH II), sepsis-related organ failure score (SOFA), perineal injury wound area (length × width/2), perineal wound depth, concomitant injury, total hospital stay, and death were collected by the electronic medical record system.

### 2.2. Types of Pelvic Fracture

The fracture types of the patients were classified according to the Tile's/AO standard, which was mainly divided into A, B, and C types. Type A (stable): type A pelvic fracture mainly involves the pubic bone and iliac crest of the pelvis and has no structural damage to the whole pelvic ring. Type A1 fracture refers to unilateral iliac crest fracture; type A2 refers to unilateral or bilateral pubic branch fracture or iliac fracture; type A3 refers to the transverse fracture of sacrum and coccyx. Type B (partially stable): type B1 fracture is mainly caused by the anterior ligament of the sacroiliac joint leading to the anterior injury of the sacroiliac joint. Type B2 is a unilateral compression injury that can lead to the ipsilateral injury of the posterior ligament of the iliac joint and anterior pubic and ischial injuries. The injury of type B3 fracture comes from the pressure on the opposite side. Type C (unstable): the injury degree of this type of pelvic fracture is more serious; it not only has rotational instability but also vertical instability. Type C1 digital sacral iliac joint was injured or dislocated. Type C2 refers to bilateral sacroiliac joint injury and even sacroiliac joint dislocation in severe cases, accompanied by the injury of the anterior pubic symphysis. Type C3 refers to sacral fractures.

### 2.3. Scoring Index

(1) GCS score: GCS score can be effectively used to judge the condition of craniocerebral injury and estimate the prognosis. The responses of eyes opening, language, and transportation were evaluated. The total score of the three items was 3–15, including mild coma (13–14 scores), moderate coma (9–12 scores), and severe coma (3–8 scores). (2) MOTS-RTS score: the score mainly includes respiratory rate, systolic blood pressure, and GCS score. Because the respiratory rate, systolic blood pressure, and the GCS score of patients can be obtained quickly in clinics, MOTS-RTS score is very operable in the treatment of acute trauma. (3) APACH II score: APACH II score is commonly used to dynamically monitor the condition of critically ill patients at present, and dynamic monitoring can more effectively predict the mortality of critically ill patients. APACH II score includes three parts: acute physiology score, age score, and chronic health score. (4) Shock index: it is used to determine whether there is shock or not or to reflect the severity of shock. Shock index = pulse rate/systolic blood pressure is calculated according to the formula to help determine the shock and the severity of shock. Shock index>1.0–1.5 indicates shock, > 2.0 indicates severe shock.

### 2.4. Statistical Analysis

SPSS20.0 and GraphPadPrism5.0 software were used for data processing. The counting data are expressed by the number of cases, and the measurement data are expressed by mean ± standard deviation. Kaplan–Meier curve was used for survival. The logarithmic rank test was used to calculate the significance of differences among subgroups. Stepwise multivariate Cox regression analysis was used to find out the independent prognostic factors related to survival. When *P* < 0.05, it was considered that the difference was statistically significant.

## 3. Experimental Results

### 3.1. Demographic Characteristics of Patients

Among the 153 patients, 94 (61.44%) were males and 59 (38.56%) were females. The average age was (43.2 ± 16.8) years, ranging from 1 to 87 years old. The cases were mainly concentrated in the two age groups of 20 to 29 years old and 50 to 59 years old, accounting for 35.29% (54/153) of all patients, as shown in Figure 1. 79 (51.63%) farmers were among the main injured group, followed by 52 (33.9%) workers. In terms of injury months, from January to December, the number of injuries were 16 (10.46%), 17 (11.11%), 8 (5.23%), 8 (5.23%), 6 (3.92%), 7 (4.58%), 8 (5.23%), 7 (4.58%), 11 (7.19%), 17 (11.11%), 23 (15.03%), and 25 (16.34%), respectively. In a year, pelvic fractures are mainly concentrated in January, February, November, and December, as shown in Figure 1. In terms of injury time, there are mainly two periods of time in a day: 10 : 00–12 : 00 and 15 : 00–18 : 00.

### 3.2. Cause of Injury of Patients

Among the 153 cases of pelvic fracture, there were 36 cases of type A fracture (23.53%), 60 cases of type B fracture (39.22%), and 57 cases of type C fracture (37.25%). The causes of injury in the whole group included traffic accident in 79 cases, fall from height in 41 cases, flat ground fall in 15 cases, accident in factory and mine in 4 cases, crush injury in 3 cases, firearm injury in 2 cases, puncture injury in 3 cases, and other 2 cases. The main cause of injury was fall injury in patients under 20 years old, traffic injury in patients aged 20 to 69 years old, and falling on the ground in people over 70 years old.  Table 1 is the comparison of the causes of injury in patients of different ages.

### 3.3. Combined Injury

Among the 153 patients, 129 cases had combined injuries, accounting for 84.31% of the total. 37 cases (19.47%) were complicated with limb fracture or ligament injury, 30 cases (15.79%) with subcutaneous hematoma, 28 cases (14.74%) with a rib fracture, 22 cases (11.58%) with hemopneumothorax, 17 cases (8.95%) with abdominal organ injury, 16 cases (8.42%) with spinal fracture, 14 cases (7.37%) with craniocerebral trauma, and 12 cases (6.32%) with urinary system injury. Extensive skin avulsion was found in 8 cases (4.21%) and sacral plexus injury or rectal injury in 6 cases (3.16%).

### 3.4. Overall Condition of Patients at the Time of Admission

The MOTS-RTS scores of the patients in the undead group and the dead group were (7.12 ± 1.52), (2.69 ± 0.96), ISS scores were (27.36 ± 15.84), (61.32 ± 7.08), GCS scores were (12.84 ± 3.69), (4.13 ± 1.25), APACH II scores were (12.87 ± 8.84), (32.41 ± 6.98), and SOFA scores were (6.68 ± 5.87), (17.12 ± 3.12). Compared with the death group, the MOTS-RTS and GCS scores of the nondeath group were significantly higher, while the ISS score, APACH II score, SOFA score, and shock index were significantly lower.  Figure 2 shows the comparison of various scores for patients with wdifferent survival statuses.

### 3.5. Treatment Methods and Complications

Among the 153 patients with pelvic fractures, 93 patients (60.78%) received nonoperative treatment and 60 patients received surgical treatment (39.22%). Of the 60 patients, 45 patients (75.00%) received open reduction and internal fixation, 10 patients (16.67%) received closed reduction and external fixator fixation, and 5 patients (8.33%) chose bone traction. There were 10 types of complications in 48 patients, including infection (*n* = 32), shock (*n* = 10), ARDS (*n* = 7), respiratory failure (*n* = 5), heart failure (*n* = 4), multiple organ failure (*n* = 3), stress ulcer (*n* = 1), diffuse intravascular coagulation (*n* = 1), and pulmonary embolism (*n* = 1).

### 3.6. Short-Term Overall Survival Rate and Cause of Death

During the hospitalization, of the 153 patients, 21 died and 122 survived, with an overall mortality rate of 13.7%. Twelve patients died in the acute stage, including 7 cases of fatal hemorrhage and 5 cases of craniocerebral injury. 9 patients died one month after hospitalization, 5 patients died of septicemia, and 4 patients died of multiple organ failures. Of the 153 patients, 21 died and 122 survived.

The average perineal trauma area of undead patients and dead patients was (54.5 ± 113.52) cm^2^ and (262.63 ± 300.84) cm^2^, respectively. The perineal trauma area of dead patients was significantly larger than that of undead patients. The average depth of perineal trauma in undead patients and dead patients was (9.63 ± 7.22) cm and (16.23 ± 10.13) cm, respectively. The survival curve showed that the larger the area of perineal injury (*c*^2^ = 5.632, *P* < 0.001) and the deeper the depth of perineal trauma (*c*^2^ = 4.897, *P* < 0.001), the lower the survival rate of patients.  Figure 3 presents survival curves for patients with different trauma depths and areas.

### 3.7. Multivariate Analysis of Patients' Prognosis

Cox multivariate analysis showed that complications, MOTS-RTS score, ISS score, GCS score, perineal trauma area, and depth of perineal trauma were independent risk factors affecting the prognosis of patients with pelvic fracture with perineal injury.  Table 2 shows Cox multivariate analysis affecting patient outcomes.

## 4. Experimental Result Analysis

In the past, most of the literature studies were reported on pelvic fracture or open pelvic fracture, but there were a few reports on pelvic fracture with perineal injury. With the development of social economy, the incidence of such injuries in China is increasing year by year [8]. Although the overall incidence of perineal injury is low, but the incidence of complications and mortality is relatively high, most patients need multidisciplinary teamwork (MDT) treatment. Generally speaking, an unstable pelvic fracture with a shock or organ injury is called a severe pelvic fracture, which can easily lead to complications such as systemic inflammatory response syndrome, fat embolism, adult respiratory distress syndrome, and multiple organ failures [9]. In patients with severe perineal laceration and severe pelvic fracture, the amount of bleeding is much larger than that of a closed fracture due to open wound. Hemorrhagic shock is the main cause of early death. The perineal wound is close to the opening of the anus, urinary tract, and vagina, and reaches the part of bone fracture, which can communicate with the pelvic cavity and abdominal cavity [10]. The wound is easily contaminated by vaginal, urethral, and anal excreta. The above factors are easy to cause pelvic abscess and peritonitis, and even serious infection of the whole body [6]. Infection is the main difficulty in the later treatment of these kind of patients. The instability of pelvic fracture can lead to secondary injury during slight movement, which increases the pain of patients and increases the difficulty of wound dressing change and daily nursing [11].

In this paper, a retrospective analysis of 153 patients with a pelvic fracture with perineal injury showed that most of the 21 dead patients had a hemorrhagic shock on admission, and 5 patients had an uncontrollable massive hemorrhage. This kind of injury is extensive, complex, and serious. It is often accompanied by abdominal, craniocerebral, and thoracic and abdominal multiple trauma, and there is a large amount of active bleeding [12]. Hemostatic techniques such as pelvic external fixator, abdominal and pelvic bandage fixation, internal iliac artery embolization, and surgical gauze packing are still difficult to control [13]. After active antishock therapy and effective hemostatic treatment, active bleeding in some patients with hemorrhagic shock can be quickly controlled and their condition can be quickly improved. Because pelvic hemorrhage usually comes from pelvic venous plexus injury, although the bleeding rate of arterial injury is small, the bleeding speed is fast, and it is difficult to stop bleeding by pressing or reducing the volume of the lumen. Most of them must be embolized by DigitM subtraction angiography (DSA) technique or ligation directly to stop bleeding [14]. Therefore, hemorrhagic shock is the main risk factor for death in patients with a pelvic fracture with perineal injury. It is suggested that the nature of bleeding should be identified as soon as possible while antishock, and effective measures should be adopted to further control active bleeding [15]. The longer the time before admission, the faster the speed of bleeding, the more serious the shock, and the lower the success rate of treatment.

For patients with a pelvic fracture with hemodynamic instability, the first priority is to quickly open venous channels and restrict fluid resuscitation against shock, and, if necessary, multichannel rapid fluid replacement and selective use of pressurized infusion device can be evaluated according to the antishock effect of fluid replacement [16]. The principle of rehydration is to start fast and then slow, with crystals first and then colloids. Appropriate transfusions of blood, haemostatic agents, and anticoagulants can improve anaemia, systemic bleeding, and coagulation. The lower the shock index, the greater the risk of death. When the symptoms and signs of early traumatic hemorrhagic shock are not obvious or in the early stage of shock, only the pulse increases, the blood pressure does not decrease obviously, or the blood pressure does not decrease but the stress increases. At this time, we need to rely on the evaluation and judgment of the injury [17]. Comprehensive assessment and analysis should be made in relation to the whole body, including expression, consciousness, mental state, skin colour, skin temperature, peripheral circulation, and urine volume. For the highly suspected manifestations of preshock or early shock, effective antishock treatment must be carried out immediately. Appropriate fluid replacement is carried out according to the principle of limited fluid resuscitation, dynamic evaluation of the patient's reactivity, possible change trend of the disease, estimation of the rate and volume of bleeding, estimation of the amount of blood preparation or transfusion needed in the later stage, and the severity of the injury [18]. The simplest method of fixation for open pelvic fractures is to wrap the pelvis with bed sheets to reduce the volume of the retroperitoneal compartment and to stop bleeding by tamponade.

This paper investigated a total of 8 causes of injury, mainly focused on traffic accidents, high fall and flat fall, and other three causes. The height fall injury of male patients is higher than that of female patients, which is related to male work and occupation, and on the one hand, high-altitude workers are mainly male patients [19]. On the other hand, women account for a higher proportion of patients who fall on the flat ground, which may be related to the fact that the severity of osteoporosis in female patients is higher than that in male patients, which is more likely to lead to low-energy pelvic fractures. There are two peaks in the incidence of pelvic fracture; the first is between 20 and 29 years old, and the level of activity in this age group is high, which is mainly caused by high-energy injuries such as car or motorcycle accidents; the second peak is in patients over the age of 50 and 59 years old. The elderly patients are prone to osteoporotic fracture due to the decrease of bone mass and bone quality, and the main patients are female patients, mostly caused by low-energy injury [20]. Traffic accidents are the main cause of pelvic fractures. Vulnerable groups such as pedestrians still have a high incidence of traffic accidents, so how to effectively improve pedestrian traffic safety and reduce the risk of pedestrian casualties is an important problem to be solved in the field of road traffic safety research. Farmers and migrant workers are the main injured patients with pelvic trauma. To adjust the rural economic structure, improve the income level of farmers, improve the concept of rural education, increase investment in rural education, and strengthen the construction of rural teachers are urgent problems to be solved.

## 5. Conclusion

In conclusion, the main causes of death of perineal trauma patients with pelvic fractures were a refractory hemorrhagic shock in the early stage and infection, septic shock, and multiple organ failure in the middle and late stages. Hemorrhagic shock in perineal trauma patients with type C pelvic fractures is difficult to control, and repeated infections and septic shock may indicate an increased risk of death. Close monitoring of bleeding, infection and shock, effective control of active bleeding, and active prevention and treatment of infection will help to reduce mortality.

## Figures and Tables

**Figure 1:** Gender distribution and injury month distribution of patients.

**Figure 2:** Comparison of various scores for patients with different survival statuses.

**Figure 3:** Survival curves for patients with different trauma depths and areas.

**Table 1:** Comparison of the causes of injury in patients of different ages.

Age	Traffic accident	Fall from height	Flat ground fall	Accident in factory	Hit injury	Crush injury	Firearm injury	Puncture injury	Other
0～9	4	11	0	0	0	0	0	0	1
10～19	3	13	0	0	0	0	0	0	0
20～29	10	4	0	2	0	2	2	0	1
30～39	14	4	0	1	3	1	0	1	0
40～49	13	3	0	1	1	0	0	2	0
50～59	17	3	0	0	0	0	0	0	0
60～69	13	1	3	0	0	0	0	0	0
70～79	3	1	5	0	0	0	0	0	0
80～89	2	0	7	0	0	0	0	0	0

**Table 2:** Cox multivariate analysis affecting patient outcomes.

Index	*β*	Se	Wald	Df	*P* Value	95% CI
Age	0.363	0.541	0.985	1	0.341	0.652～2.632
Gender	0.287	0.369	0.254	1	0.896	0.142～1.874
Classification of fracture	0.869	0.326	1.133	1	0.259	1.261～4.502
Complication	0.678	0.335	4.078	1	0.041	1.021～3.980
MOTS-RTS score	0.189	0.268	8.464	1	0.009	0.495～1.398
ISS score	0.523	0.296	2.181	1	0.038	0.951～2.993
GCS score	0.452	0.166	2.632	1	0.030	0.864～3.336
APACH II score	0.240	0.263	0.830	1	0.369	0.472～1.318
SOFA score	0.359	0.523	0.512	1	0.636	0.538～3.815
Perineal trauma area	0.852	0.352	7.174	1	0.010	1.264～4.564
Depth of perineal trauma	0.239	0.213	11.154	1	<0.001	0.787～1.874

## Data Availability

The simulation experiment data used to support the findings of this paper are available from the corresponding author upon request.
